# Hematological reference intervals for adult population of Dire Dawa town, East Ethiopia

**DOI:** 10.1371/journal.pone.0244314

**Published:** 2021-02-16

**Authors:** Teklay Mengistu Sissay, Melatwork Tibebu, Tagesachew Wasihun, Aster Tsegaye

**Affiliations:** 1 Dil Chora Hospital, Dire Dawa, Ethiopia; 2 Department of Medical Laboratory Sciences, College of Health Sciences, Addis Ababa University, Addis Ababa, Ethiopia; University of Mississippi Medical Center, UNITED STATES

## Abstract

**Background:**

Reference interval (RI) for hematological parameters is used to interpret laboratory test results in the diagnosis, management and monitoring of hematologic disorders. Several factors including sex, age, dietary patterns, pregnancy status, ethnicity and geographic location affect hematological RIs. However, manufacturers derived reference value is currently in use in most developing countries including Ethiopia. This study aimed to establish hematological RIs for adult population living in Dire Dawa town, East Ethiopia.

**Methods:**

In this cross-sectional study, 513 apparently healthy adults of Dire Dawa town were enrolled from January to March 2019. From these, 342 (171 males and 171 non-pregnant females) were aged 18–65 years while 171 were pregnant women aged 15–49 years. After obtaining written informed consent, 5ml fresh whole blood was collected of which 2ml was used for hematologic analysis using Mindray BC-3000plus hematology analyzer and 3ml for serological tests. The 2.5^th^ and 97.5^th^ RI was computed by non-parametric test employing SPSS version 24. P-value <0.05 was considered statistically significant.

**Result:**

Males had significantly higher reference value for most of red cell parameters (Hgb, RBC, HCT, MCH and MCHC) than females (p <0.05), while most of the WBC parameters were significantly higher in females than males. Moreover, non-pregnant women had higher values for most of red cell parameters than pregnant women. Pregnant women had higher WBC parameters than their non-pregnant counterparts.

**Conclusion:**

The hematologic RIs obtained in this study shows variation between genders, between pregnant and non-pregnant women, from the clinical practice currently utilised in Dire Dawa town and from studies conducted in Ethiopia, African countries as well as the Western population. It underscores the need for utilising gender and pregnancy specific, locally derived hematologic RI for better management, diagnosis and monitoring of hematologic disorders for adults of both genders and pregnant women.

## Background

Reference intervals (RIs) are used for a comparative decision-making process by describing the typical distribution of results derived from healthy reference population. The values aid in the interpretation of clinical laboratory results for patient care in the diagnosis, therapeutic management and other physiological assessment [1, 2] including for recruitment of participants in clinical trials. The complete blood count (CBC) is the most frequently requested clinical laboratory test to establish diagnosis, management, monitoring of hematologic disorders and other medical problems [3].

Hematologic result interpretation relies on the RI derived from healthy individuals representing the population to be served [3]. Gender, age, genetics, dietary patterns, pregnancy, ethnic origin and prior exposure to environmental pathogens are among factors affecting hematologic RIs [4, 5]. These factors preclude the use of RIs determined even within the same country of diverse population groups. Although age and sex are the two most common RIs partitioning criteria, hematologic variations are also indicated during pregnancy. In order to nurture and accommodate the developing foetus, pregnancy is characterized by many physiological and hematological changes, which may appear to be pathological in the non-pregnant state [6, 7].

Only minority of clinical laboratories are sufficiently resourced in terms of time, finance and expertise to establish RIs for all, or indeed any of the tests they routinely perform [8]. As a result, reference values currently in-use by many laboratories of developing countries are provided by companies and Dire Dawa town is not an exception in this regard. Adopting reference values derived from dissimilar population source without consideration of local differences may lead to misdiagnosis and misclassification of disease, increase cost by unnecessary investigations and risk in patient safety as well. Therefore, this study was carried out to determine hematological parameters RIs of apparently healthy adults of Dire Dawa population by applying the classical and advanced statistical methods recommended by Clinical Laboratory Standard Institute (CLSI) [9]. Ethiopia having a diverse population groups, the determination of RI for Dire Dawa population will add to the existing body of information from the other parts of the country, while specifically serving the clinical management of the town residents.

## Materials and methods

### Study design, area and setting

A cross sectional study was carried out in Dire Dawa City Administration (DDCA), East Ethiopia from January to March 2019. DDCA is the second chartered city of Ethiopia, which is located 515 kilometres away from the capital city Addis Ababa. It is geographically located between 9^o^49 North latitude and 42^o^19 East longitude at an altitude ranging from 950–2260 (an average of 1160) meter above sea level. Dire Dawa has a hot and dry climate with an average temperature of 24.6°C. Based on the 2007 national census report of Central Statistical Agency of Ethiopia, DDCA has a total population of 384,000, of whom the majority (74%) of people live in urban area.

### Population

Participants included in this study were apparently healthy adults of both sexes and pregnant women. Written informed consent was obtained from each participant after explaining the purpose, risks and benefits of the study. Volunteers were interviewed face-to-face using a pre-tested and semi-structured questionnaire to gather information on demographic data, clinical and medical history, health condition, risk factors and life styles. Vital sign assessment (body temperature, body weight, blood pressure and pulse rate) using digital devices and physical examinations were performed by clinicians. All participants were screened for HIV, Hepatitis B surface antigen (HBsAg), Hepatitis C antibody (HCV-Ab), *Treponema pallidum*. C-Reactive Protein (CRP), which is an acute phase reactant protein produced and secreted by the liver in response to any inflammation in the body, was measured using a qualitative test. Moreover, malaria screening of all participants and pregnancy test to females were also performed.

### Inclusion criteria

Inclusion into the study was based on the following criteria: aged 18–65 years for adults and 15–49 for pregnant women; presenting a written signed consent; volunteer to provide whole blood and urine sample (for females); resided in Dire Dawa town for at least five years; subjectively feel healthy and having normal records of vital sign and physical examination.

### Exclusion criteria

- Individuals were excluded prior to blood withdrawal if he or she was with at least one of the following known diseases like: hypertension, diabetes mellitus, chronic gastritis, cancer, cardiac illness, bleeding disorders, allergy, anemia, and any unspecified chronic diseases.
- Individuals with history of blood transfusion within the last one year or donated blood within the last six months, hospital admission for the last one year, had surgery in the last three years, had malaria in the last six months, and diagnosed with any form of tuberculosis in the last two years.
- Individuals who were drug abusers, had work exposure to hazardous chemicals, smokers, and more than occasional (holidays, special ceremonies) alcohol drinkers and Khat (*Catha edulis*) chewers. Khat is a plant with a natural distribution in the Eastern part of Ethiopia and its chronic use is associated with the development of several systemic and metabolic disorders.
- Moreover, pregnant women with active bleeding during the data collection period encountered pregnancy and obstetrics complication; and non-pregnant women who were menstruating during the data collection period; whose average menstruation stay >7days; or have taken over the counter of oral contraceptive and are breast feeding were also excluded from the study.

### Sample size and sampling strategies

The sample size was determined based on the CLSI recommendation [9], which states a minimum of 120 participants are required from each partition for RI determination. In this study, by considering the CLSI recommendation additional 30% rejection rate for transfusion transmittable infections (HIV; Hepatitis B and C; Syphilis; and malaria) and inflammation which was taken from previous study conducted in Africa [10] was taken into account to determine the total sample size per group. Accordingly, a total of 513 participants (171 from each partition) were recruited by a priori sampling method using a well-defined inclusion and exclusion criteria.

To recruit adult study participants of both sexes from the community, three of the nine urban kebeles, which is the smallest administration unit, and eight of the thirty-eight rural kebeles were selected randomly by considering population distribution. Health extension workers recruited participants from the community of selected kebeles, while clinical nurses recruited pregnant women from the antenatal clinic (ANC) of Dil Chora Hospital, conveniently.

### Sample collection

Five-millilitre venous blood was collected from antecubital vein under aseptic conditions between 08:00 a.m. and 11:00 a.m. from eligible study participants, who fasted for at least 8 hours. Participants were in a sitting position for at least 15 minutes before blood collection. Two ml whole blood were dispensed into Dipotassium Ethylene Diaminetetraacetic acid (K_2_EDTA) Vacutainer tube (Becton Dickinson, Franklin Lakes, NJ, USA) for hematologic analysis while the remaining 3ml was dispensed into plane tube and centrifuged (3,000 rpm, 15minutes) within two hours of sample collection for serologic tests. Urine sample was collected from non-pregnant women, to rule out pregnancy, using leak free clean container. All samples were labelled, placed in separate and sealed sample transporting container and shipped at room temperature to DCH laboratory within one hour after collection.

### Laboratory assays

The whole blood samples were analysed within two hours after blood drawing using Mindray BC-3000 Plus automated hematology analyzer (Mindray Bio-medical electronics Co., Ltd., Shenzhen, China), which performs 18 hematologic parameters, for *in vitro* diagnosis use in clinical laboratories. The measured parameters were white blood cell count (WBC), granulocyte count (Gran#), lymphocyte count (Lymph#), mixed cells count (MID#), granulocyte percentages (Gran%), lymphocyte percentages (Lymph%), mixed cells percentages (MID%), red blood cell (RBC) count, hemoglobin (Hgb), hematocrit (HCT), mean corpuscular volume (MCV), mean corpuscular hemoglobin (MCH), mean corpuscular hemoglobin concentration (MCHC), red cell distribution width (RDW), platelets count (PLT), mean platelet volume (MPV) and platelet distribution width (PDW).

The analyser uses electrical impedance method for cell counting and cyanide free method for hemoglobin determination. Well-trained laboratory staffs performed all experiments according to the Dil Chora Hospital laboratory standard operating procedures (SOPs).

Serological tests were determined on serum samples using the following commercially approved rapid test kits: HIV1/2 STAT-PACK (Chembio Diagnostics System, Inc. USA.), HBsAg (Acon Laboratories, Inc. USA), HCV-Ab (Henso Medical (Hangzhou) Co., Ltd, China), *Treponema pallidum* (ENTEROCHECK-WB, Zephyr Biomedicals, A Division of Tulip Diagnostics (P) Ltd, India) were used to screen for HIV, HBV, HCV and syphilis respectively. CRP was determined using HumaTex RF (Human Diagnostics, Worldwide). A one-step qualitative pregnancy test was performed for the presence of β-HCG (Laboquick HCG strip, Korglu Ltd, Turkey) using urine sample. Both thin and thick blood smears were made directly after collection of blood, air-dried, fixed (for thin smear) and stained with Giemsa stain for malaria screening.

### Quality control

All laboratory procedures were performed based on the Dil Chora Hospital Laboratory SOPs and according to the manufacturers’ recommendations. Prior to tests, each day internal quality control (QC) was performed using three level (low, normal and high) commercial quality control material and the analyzer was calibrated as per the manufacturer recommendation. All the daily quality control runs were plotted on LJ charts and results of all hematolologic parameters were within ± 2 SD from their target values. Our laboratory is enrolled in the one world accuracy proficiency programs for hematology analysis and it had satisfactory performance for all hematologic parameters processed over the study period. Moreover, between-run precision was assessed for 20 consecutive days by each internal QC material. The mean, standard deviation (SD) and coefficient of variation (CV) were calculated. Each CV was compared against the values given in the analyser manual and it was within the manufacturer acceptable limit.

### Statistical analysis

Data was cleaned, edited, checked for completeness manually and entered daily using IBM-SPSS Version 24 statistical software (SPSS version 24.0, SPSS Inc. Chicago, IL, USA) for analysis. RI was determined by calculating the 2.5^th^ and 97.5^th^ percentiles based on the CLSI guideline [9]. The Dixon method was used to check for outliers and the Kolmogorov-Smirnov tests were used to assess normality of the data distribution. Based on the data distribution, effect of gender was compared using the Mann-Whitney U test and independent-sample t-test while trimester specific variations among pregnant women were evaluated by one-way ANOVA and Kruskal Wallis test. The proportion of Out of Range (OOR) values was also calculated to evaluate the current clinical practice of utilizing reference value in different laboratories found in Dire Dawa town against the RIs generated by our study. A two-sided *p value* < 0.05 was considered statistically significant.

### Ethics approval and consent to participate

The study was conducted after the study protocol was reviewed and approved by the Departmental Research and Ethics Committee of the Department of Medical Laboratory Sciences, College of Health Science of Addis Ababa University. Moreover, official letter of permission was obtained from Dire Dawa Regional Health Bureau. Informed written consent was also obtained from each study participant prior to data collection. Participants positive for any of the tests were linked to health facilities by providing them the test results.

## Results

### Demographic and clinical characteristics

A total of 513 individuals were enrolled in this study with equal number of participants from each partition (171 each males, non-pregnant females and pregnant-women). Among these individuals, 41 (8%) were excluded from analysis due to being positive for HIV (6, 14.6%), HBsAg (12, 29.2%), Syphilis (2, 4.9%) and positive for CRP (23, 56.1%). Among the excluded, two participants were positive for both HIV and CRP (hence making the sum 43). After exclusion of data for positive participants, no additional outliers were identified. The remaining 472 participants (160 males, 155 females and 157 pregnant women) were deemed healthy and included in the final analysis. The age distribution for each study group are shown on Fig 1. The median age for adult males, adult females and pregnant women were 32 years [IQR: 27–41 years], 31 years [IQR: 24–39 years], and 26 years [IQR: 23–28 years], respectively. Of the total 157 pregnant women, 42(26.8%), 50(31.8%) and 65(41.4%) were in first (1–12 weeks of gestation), second (13–27 weeks of gestation) and third trimester (28–40 weeks of gestation), respectively.

**Fig 1:** Age distribution histogram of study participants.

### Hematological parameters reference intervals

Table 1 show the calculated median and 95% RI (2.5^th^-97.5^th^ limits) for the hematologic parameters of the three study groups.

**Table 1:** Median and 95% RI values of WBC, RBC and platelet parameters of adult males, adult females and pregnant women of Dire Dawa population, Ethiopia from January-March, 2019.

Parameter	Category	N	Median	RI (2.5^th^-97.5^th^)	90% CI		P-value	
					LLC	ULC	M & F	NP & P
**WBC (x10**^**9**^**/L)**	Male	158	5.9	3.5–10.31	3.5–3.8	9.6–10.5	^**a**^0.006*	
	Female	150	6.8	3.8–10.2	3.7–4.2	9.9–10.5		^**b**^ < 0.001*
	Pregnant	151	7.8	3.6–11.8	3.5–4.6	11.0–11.8		
**Lymph# (x10**^**9**^**/L)**	Male	157	2.1	1.2–3.81	1.0–1.4	3.3–4.10	^**a**^0.029*	
	Female	149	2.3	1.3–4.03	1.2–1.4	3.5–4.2		^**a**^< 0.001*
	Pregnant	151	1.9	1.1–2.62	1.0–1.2	2.4–2.8		
**Gran# (x10**^**9**^**/L)**	Male	159	3.3	1.4–6.8	1.2–1.5	6.3–7.1	^**a**^0.003*	
	Female	151	3.9	1.4–7.0	1.1–1.8	6.5–7.1		^**b**^< 0.001*
	Pregnant	151	5.4	2.3–9.12	2.1–2.8	8.3–9.6		
**Lymph%**	Male	157	36.6	18.2–54.8	17.9–20.8	52.5–56.9	^**a**^0.098	
	Female	152	34.3	18.1–55.1	17.7–20.8	55.1–57.5		^**a**^< 0.001*
	Pregnant	151	23.5	14.0–39.6	13.3–15.4	36.6–40.5		
**Gran%**	Male	156	52.6	33.1–72.8	28.5–36.7	69.0–75.4	^**a**^0.042*	
	Female	147	57.1	39.9–71.2	33.5–39.9	69.7–72.5		^**a**^< 0.001*
	Pregnant	152	67.7	49.3–79.8	48.7–52.6	78.8–80.7		
**Hgb (g/dL)**	Male	158	15.2	12.4–17.5	11.4–13.3	17.1–17.60	^**a**^< 0.001 *	
	Female	152	12.8	10.7–15.2	10.2–11.1	14.9–15.6		^**a**^< 0.001*
	Pregnant	145	11.7	9.5–13.50	9.4–9.90	13.2–13.8		
**RBC# (x10**^**12**^**/L)**	Male	154	5.39	4.46–6.15	4.05–4.69	6.07–6.22	^**b**^< 0.001*	
	Female	149	4.73	3.81–5.49	3.75–4.06	5.43–5.65		^**b**^< 0.001*
	Pregnant	149	4.19	3.67–5.07	3.33–3.49	54.98–5.19		
**HCT (%)**	Male	159	51.3	43.8–58.5	42.6–44.8	57.70–60.6	^**a**^< 0.001*	
	Female	151	44.8	37.4–52.0	35.5–38.8	50.8–52.7		^**b**^< 0.001*
	Pregnant	148	39.2	32.2–46.0	30.5–34.2	45.3–46.8		
**MCV (fl)**	Male	150	94.2	86.3–104.4	85.1–88.8	102–105.4	^**b**^ 0.854	
	Female	141	94.7	83.4–104.2	81.3–86.5	102.7–105.7		^**b**^0.479
	Pregnant	147	94.4	84.7–103.4	82.7–86.0	101.7–104.7		
**MCH (pg)**	Male	153	27.8	24.6–31.1	24.1–25.7	30.6–31.6	^**b**^< 0.001*	
	Female	143	27.3	23.0–30.1	22.1–24.1	29.3–32.2		^**a**^0.001*
	Pregnant	147	27.6	23.7–32.6	23.1–24.2	31.7–32.8		
**MCHC (g/dl)**	Male	155	29.5	27.6–30.8	27.2–28.0	30.7–31.2	^**a**^< 0.001*	
	Female	150	28.7	26.7–29.9	26.1–27.2	29.6–30.3		^**b**^0.008*
	Pregnant	148	29.1	27.4–33.2	27.0–27.8	32.7–33.5		
**RDW-CV (%)**	Male	153	13.6	12.3–15.3	12.3–12.5	15.1–15.9	^**a**^0.883	
	Female	143	13.6	12.4–15.7	12.1–12.6	15.0–15.8		^**b**^ < 0.001
	Pregnant	148	14.0	12.5–17.6	1.40–12.7	16.7–18.2		
**RDW-SD**	Male	153	49.8	42.1–61.3	41.5–43.1	58.1–63.1	^**b**^0.003*	
	Female	146	51.4	43.1–60.9	41.5–44.8	58.4–62.3		^**a**^0.037*
	Pregnant	150	50.6	40.6–60.6	39.0–43.1	58.1–60.6		
**Platelet (x10**^**9**^**/L)**	Male	155	279	164–447	137–189	410–466	^**a**^0.004*	
	Female	148	310	177–442	144–213	405–482		^**a**^< 0.001*
	Pregnant	149	276	157–421	140–178	387–445		
**MPV (fl)**	Male	158	9.1	7.7–10.9	7.40–7.8	10.6–11.1	^**a**^0.476	
	Female	151	8.9	7.3–10.6	77.1–7.6	10.4–10.8		^**b**^ 0.833
	Pregnant	152	8.9	7.6–10.30	7.5–8.0	10.0–10.5		
**PDW (%)**	Male	152	15.6	15.0–16.3	15.0–15.1	16.1–16.5	^**a**^0.003*	
	Female	153	15.5	15.0–16.2	14.9–15.1	16.0–16.2		^**a**^< 0.001*
	Pregnant	153	15.9	15.1–16.6	14.9–15.3	16.5–16.6		
**PCT (%)**	Male	155	0.254	0.15–0.36	0.13–0.17	0.35–0.37	^**a**^< 0.001*	
	Female	147	0.280	0.18–0.38	0.14–0.20	0.37–0.39		^**b**^< 0.001*
	Pregnant	149	0.252	0.15–0.35	0.14–0.17	0.33–0.39		

LLC, Lower Limit Confidence interval; ULC, Upper Limit Confidence interval; M, Male; F, Female; NP, Non-Pregnant; P, Pregnant.

^**a**^Mann-Whitney U Test

^**b**^ independent sample t-test

*p values<0.05: statistically significant difference.

### WBC parameters reference intervals

Table 1 displays the median, 95% RI with 90% confidence interval of the lower 2.5^th^ and upper 97.5^th^ limits for WBC parameters. Females tended to have significantly higher median values compared to males for WBC counts [6.8(3.8–10.2)*10^9^/L Vs 5.9(3.5–10.3)*10^9^/L, p = 0.006]; Lymph# [2.3(1.3–4.0)*10^9^/L Vs 2.1 (1.2–3.8)*10^9^/L, p = 0.029]; Gran# [3.9(1.4–7.0)*10^9^/L Vs 3.3(1.4–6.8)*10^9^/L, p = 0.003] and Gran%[57.1(39.9–71.2)% Vs 52.6(33.1–72.8)%, p = 0.042]. However, the median MID% [9.5(5.1–13.9)% Vs 8.3(4.7–13.1)%, p = 0.001] was significantly higher in males than females. When compared between pregnant and non-pregnant females, significantly higher median WBC count, Gran# and Gran% were seen in pregnant women than non-pregnant (P = 0.001), while non-pregnant females had significantly higher Lymph# and Lymph% than pregnant women (Table 1).

### RBC parameters reference intervals

Table 1 summarizes the median, 95% RI with 90% confidence interval of the lower 2.5^th^ and upper 97.5^th^ limits for RBC parameters. In this study, significantly higher median values were noted in males for most of red cell parameters (RBC count, Hgb, HCT, MCH and MCHC) than females, while females had higher median value for RDW-SD than males as shown in Table 1. Significantly higher median values in non-pregnant women than pregnant were seen for Hgb[12.8(10.7–15.2)g/dL Vs 11.7(9.5–13.5)g/dL, p = < 0.001]; RBC count[4.73(3.81–5.49)*10^12^/L Vs 4.19(3.67–5.07)*10^12^/L, p = < 0.001]; HCT[44.8(37.4–52.0)% Vs 39.2(32.2–46.0)%, p = < 0.001] and RDW-SD[51.4(43.1–60.9) Vs 50.6(40.6–60.6)%, p = 0.037]. Pregnant females, on the other hand, had higher median values than non-pregnant for MCH [27.6(23.7–32.6)pg Vs 27.3(23.0–30.1)pg, p = 0.001]; MCHC[29.1(27.4–33.2)g/L Vs 28.7(26.7–29.9)g/L, p = 0.008) and RDW-CV [14.0(12.5–17.6)% Vs 13.6(12.4–15.7)%, p = < 0.001).

### Platelet parameters reference intervals

The median, 95% RI with 90% confidence interval of the lower 2.5^th^ and upper 97.5^th^ limits for PLT parameters are shown in Table 1. The study revealed significantly higher median vales in females than males for PLT count [310(177–442)*10^9^/L Vs 279(164–447)*10^9^/L, p = 0.004] and PCT [0.28(0.18–0.38)% Vs 0.25(0.15–0.36)%, p = < 0.001], while significantly higher median values in males than females was observed for PDW [15.6(15.0–16.3)% Vs 15.5(15.0–16.2)%, p = 0.003]. As illustrated in Table 1, significantly higher median values in non-pregnant than pregnant females were noted for PLT# and Plateletcrit (PCT) which is a measure of total platelet mass, while pregnant women had significantly higher median platelet distribution width (PDW) value than non-pregnant women.

### Hematological parameter of pregnant women based on trimesters

To illustrate the difference in hematological parameters by gestational age of pregnant women, box and whisker plots are shown for WBC count, RBC count, Hgb and platelet count (Fig 2A–2D).

**Fig 2:** Box and whisker plots showing the comparison of selected hematologic parameters (A: WBC count (x10^9^/L), B: RBC count (x10^12^/L, C: Hgb (g/dL), D: PLT count (x10^9^/L)) by gestational age among pregnant women (n: 1^st^ trimester = 48, 2^nd^ trimester = 56, 3^rd^ trimester = 53) in Dire Dawa town, Ethiopia from January-March, 2019.

A decreased trend in the median value of WBC count (Fig 2A) was observed from the 1^st^ to 2^nd^ trimester, but increased from the 1^st^ to 3^rd^ trimester [1^st^ = 7.7(2.8–12.0)*10^9^/L; 2^nd^ = 7.4(3.3–11.7)*10^9^/L and 3^rd^ = 8.0(4.1–12.0)*10^9^/L]. But there was no statistically significant difference between trimesters (p: 1^st^ & 3^rd^ = 0.229; 1^st^& 2^nd^ = 0.375 and 2^nd^ & 3^rd^ = 0.811). The RBC count (Fig 2B) decreased from the 1^st^ to 3^rd^ trimester [1^st^ = 4.38(3.65–5.21)*10^12^/L; 2^nd^ = 4.08(3.19–5.02)*10^12^/L and 4.09(3.22–4.98)*10^12^/L] with no significant difference between trimesters (p>0.05).

Significantly decreased median value of Hgb (Fig 2C) was detected from 1^st^ [(12.0(9.7–14.0)g/dL] to 2^nd^ trimester [11.4(9.2–13.2g/dL)] with p = 0.007 and from 1^st^ to 3^rd^ trimester 11.8(10.0–13.3)g/dL with p = 0.042, but no significant difference was observed between the 2^nd^ and 3^rd^ trimester (p = 0.339). The platelet count (Fig 2D) significantly decreased from the 1^st^[304 (185–404)*10^9^/L] to 2^nd^ trimester [268(137–430)*10^9^/L] with p = 0.005 and from the 1^st^ to 3^rd^ trimester [267(133–404)*10^9^/L] with p = 0.038.

### Comparison of RIs established in this study with the current practice and other studies

The study calculated the percentage for out-of range (% OOR) values, by comparing the RIs established in the current study with the company derived RIs which is currently being used in Dil Chora hospital and other health facilities in Dire Dawa town having similar equipment platform. Based on the locally derived RI in the current study, the %OOR values are displayed in Table 2. Accordingly, Hgb, 16% in males and 7.2% in females; RBC count, 8.4% in males and 6.0% in females; WBC count, 10.7% in males and 12% in females; platelet count, 17.4% in males and 22.9% in females were misclassified as having normal or abnormal values.

**Table 2:** Comparison of adult hematological reference values obtained in this study versus currently practiced RI and other studies.

Parameter	Sex	This study		The current practice		African studies							
		N	RI	RI	% Out of range	N	Ghana (15)	N	Zimbabwe (13)	N	Mali (14)	N	Asmara (18)
**Hgb (g/dL)**	Male	158	12.4–17.5	11–17	16.4%(26/158)	316	11.3–16.4	412	13.2–18.3	173	12.4–17.6	295	12.6–17.8
	Female	152	10.7–15.2	11–17	7.2%(9/152)	308	9.8–16.0	357	10.2–15.9	40	12.0–14.9	296	12.5–17.6
**RBC (x10**^**12**^**/L)**	Male	154	4.46–6.15	3.5–5.50	8.4%(13/154)	316	3.79–5.96	412	4.4–6.7	173	4.1–6.2	295	4.2–6.07
	Female	149	3.81–5.49	3.5–5.50	6.0%(9/149)	307	3.09–5.30	357	3.9–5.9	40	3.9–5.7	296	4.0–5.7
**HCT (%)**	Male	159	43.8–58.5	NA	NA	316	33.2–50.5	412	42.0–55.1	173	33.2–54.6	295	40.5–55
	Female	151	37.7–52.0	NA	NA	309	26.4–45	357	33.9–48.7	40	26.8–52.5	296	37.9–52
**MCV (fL)**	Male	150	86–104	80–100	10% (15/150)	316	70–98	412	72.8–102.6	173	72.3–97.7	295	85.7–100
	Female	141	83–104	80–100	9.1% (13/143)	309	73–96	357	68.8–100.7	40	79–118	296	85.5–100
**MCH (pg)**	Male	153	24.6–31.1	27–34	21.3% (33/155)	316	22.7–33.5	412	22.9–33.5	173	22.8–33.7	295	28–33
	Female	143	23.0–30.1	27–34	44.0% (63/143)	307	22.3–33.6	357	20.7–32.1	40	23.1–34.8	296	26.5–32.6
**MCHC (g/L)**	Male	155	27.6–30.0	32–36	50% (76/150)	315	30.6–36.0	412	29.8–35.4	173	30.9–34.9	295	30.4–33.7
	Female	150	26.7–29.9	32–36	60.6 (91/150)	305	30.4–36.5	357	29.2–34.3	40	30.9–34.5	296	30–33.7
**WBC (x10**^**9**^**/L)**	Male	158	3.5–10.3	4–10	10.7 (17/158)	311	3.5–9.2	412	2.8–8.1	173	3.7–11.1	295	3.7–9.3
	Female	150	3.8–10.2	4–10	12% (18/150)	309	3.5–9.2	357	3.3–8.3	40	3.8–12.5	296	3.3–8.9
**Gran# (x10**^**9**^**/L)**	Male	159	1.4–6.8	2.0–7.0	15.7% (25/159)	313	1.5–5.9	412	0.77–3.9	173	1.0–4.4	295	NA
	Female	151	1.4–7.0	2.0–7.0	10% (15/151)	309	1.4–5.5	357	1.1–4.4	40	1.2–7.4	296	NA
**Lymph#(x10**^**9**^**/L)**	Male	157	1.2–3.8	0.8–4.0	2.5% (4/157)	316	1.2–5.2	412	1.1–3.2	173	1.2–3.8	295	NA
	Female	149	1.3–4.0	0.8–4.0	4.0% (6/149)	308	1.2–4.4	357	1.3–3.7	40	1.4–4.6	296	NA
**Gran (%)**	Male	156	33.1–72.8	50–70	44.8% (70/156)	316	30.2–69.9	412	22.1–62.8	173	26–66	295	31.7–73.6
	Female	147	39.9–71.2	50–70	34.0% (50/147)	309	33.3–67.5	357	27.1–62.0	40	26–67	296	33.5–70.5
**Lymph (%)**	Male	157	18.2–54.8	20–40	36.9% (58/157)	315	24.0–57.2	412	24.1–60.3	173	NA	295	22–59.9
	Female	152	18.1–55.1	20–40	32.8% (50/152)	309	26.9–58.3	357	28.4–59.0	40	NA	296	22.3–58.2
**PLT (x10**^**9**^**/L)**	Male	155	164–447	100–350	17.4% (27/155)	316	88–352	412	125–357	173	133–460	295	128–318.6
	Female	148	177–442	100–350	22.9% (38/148)	309	89–403	357	163–431	40	151–460	296	145–351

**Ghana**, age: 18–59 years, author: *Dosoo DK*, *et*.*al*. Year: 2012; **Zimbabwe**: age: 18–55, author: *Samaneka WP*, *et*.*al*. Year: 2016; **Mali**, age: 18–59 years, author: *Kone B*, *et*.al. Year: 2017 **Asmara**, age: 18–49 years, author: *Siraj N*, *et*.*al*. Year: 2018. *RI*, *Reference Interval; WBC#*, *White Blood Cells; LYM#*, *Lymphocytes counts; Gran#*, *Granulocytes count; MID#*, *Mixed Cells count; RBC*, *Red Blood Cell count; Hgb*, *Hemoglobin; HCT*, *Hematocrit; MCV*, *Mean Corpuscular Volume; MCH*, *Mean Corpuscular Hemoglobin; MCHC*, *Mean Corpuscular Hemoglobin Concentration; PLT#*, *Platelet Count*.

The study also tried to compare the current RIs with studies from different geographic location of Africa like Asmara, Ghana, Mali and Zimbabwe. As seen in Table 2, this study illustrated that the RIs determined are only partly comparable to others and no consistent pattern is seen in the reports from the different countries. Of note, the finding of low WBC lower limit seems universal across the studies though values vary. On the other hand, the lower limit for PLT in the current study is higher than the limits from Asmara, Ghana and Zimbabwe.

## Discussion

This study is the first of its kind conducted in the Eastern part of the country, which aimed to establish hematological parameter reference intervals of Dire Dawa population. The study involves adult male, female and pregnant women.

The current study confirmed earlier findings that males had significantly higher values for most of RBC parameters (Hgb, HCT, RBC, MCH and MCHC) than females [11–16]. This could be explained on the basis of the effect of sex hormones, both estrogen and androgens, on erythropoiesis and the lower iron storage in females because of iron losses during regular menstruation [17].

This study illustrated that the RI determined is only partly comparable with some of the hematologic parameters reported by African literatures. For instance, comparable RI was found between this study and a study from Asmara for RBCs count, HCT and Hgb (males) [18]. This could partly be due to the genetic similarity that both Dire Dawa and Asmara population were the same nation before Eritrean independency from Ethiopia. Moreover, except for the lower Hgb values of the lower reference limit of females, comparable RBC count and Hgb RI was also indicated in a study from Mali [14]. However, our study RI is higher than the Ghanaian for Hgb, RBCs and HCT; and lower than Zimbabwean males for Hgb and RBC count [13, 15]. This variation for the red cell parameters could be attributed to the difference in the socio demographic, dietary and genetic factors among different populations. Methodological variations among the different studies could partly explain the observed differences.

Most of the red cell parameters (RBC count, Hgb and HCT) RIs from different parts of Ethiopia are higher than our study RIs in both genders [19–23]. This inconsistency may be due to the geographical location differences that Dire Dawa is located at lower altitude than the studies conducted in the northern part of Ethiopia like Debre Markos (altitude, 1800 m), Gondar (altitude, 2200 m), Bahir Dar Town (altitude, 1,830 m), Addis Ababa (altitude, 2,355 m), and South west Ethiopia (altitude, 1788 m) [19–23]. In order to compensate for the low partial pressure of oxygen at high altitude, Hypoxia Inducible Factor-1 (HIF-1) alpha, erythropoietin and RBC in the acclimatisation process, together with the fall in plasma volume increases the concentration of hemoglobin in the early stages of hypoxic exposure [24]. This indicates the need to define population specific RI, given the potential differences among distinct geographical regions even in the same countries. Cultural differences in dietary habit exist between the northern and eastern part of Ethiopia as well as among African countries. *Teff*, a tiny grain that is rich in iron is a staple diet in the northern part of Ethiopia while sorghum and maize are widely used in the eastern part of Ethiopia. Such dietary pattern differences could possibly contribute to the observed differences and also justify the need for population specific RIs for hematological parameters.

We also found higher median WBC count in females than males (6.8 vs 5.9x10^9^/L)which is consistent with a report from southern Taiwan [25]. On the other hand, the RI for WBC count is comparable with studies conducted in Ethiopia, like Debremarkos and Bahdar [19, 22]; however, differences was noted in comparison to studies conducted in Southwest Ethiopia [20], The observed differences could be attributed to methodological differences to some extent although differences in prevalence of infections among the different populations cannot be ruled out. The current study, however, has used stringent exclusion criteria both at enrolment and during data analysis.

Significantly higher PLT count in females than males (310 vs 279 x10^9^/L) in our study is consistent with previous reports from Oman, Thailand, Zimbabwe and Mali [11–14]; and studies conducted in Ethiopia [19, 20, 26]. Females have lower total body iron storage but higher estrogen level, which favours stimulation of higher platelet production than males [25]. This suggests the need for utilizing gender specific hematologic RI for result interpretation to aid accurate diagnosis of disease, decrease patient suffering from progress of disease and reduce unnecessary costs.

In both sexes, the upper and lower limit for the PLT count RI in the current study is higher than those reported from other African studies [13, 15, 18] and United States [27]. Evidences indicated that there is a micro-heterogeneity in platelet parameters even among ethnically homogeneous subjects living in the same country and region as well [28].

Another important finding of significantly higher median WBC count (7.8 vs 6.8 x10^9^/L) and Gran# (5.4 vs 3.9 x10^9^/L) but lower PLT (276 vs 310 x10^9^/L) count, Hgb (11.7 vs 12.8 gm/dL) and Lymph# (1.9 vs 2.3 x10^9^/L) in the pregnant than the non-pregnant females is consistent with studies reported from Beijing and Nigeria [29, 30]. The lower values for most of RBC parameters in the pregnant than non-pregnant women are expected physiological changes. During pregnancy there is an increase in plasma volume in response to an under-filled vascular system as well as an increased iron demand for the developing fetus which results in decreased Hgb, HCT and RBC count [31].

On the contrary, leucocytosis occurring in pregnant women than the non-pregnant is an indication for adequate bone marrow response to an increased drive for erythropoiesis. Evidence indicated that by 4 weeks post-delivery, the WBC RI become similar to those in healthy non-pregnant women [31]. The lower Lymph# and Lymph% while higher Gran# and Gran% in pregnant women than the non-pregnant are attributed to the progressive elevation of the innate immune system and suppression of the adaptive immune system during pregnancy [32].

The lower PLT count in pregnant than non-pregnant could be during pregnancy there is an increased consumption of PLT as well as decreased life span in the utero placental circulation [7]. This is also supported by the observation that during post-delivery the PLT count increases in reaction to and as a compensation for increased PLT consumption during the process of delivery [31].

The current study compared the pregnant women data by trimester. The increase in the median value of WBC count from the first to third trimester of our study is consistent with other findings [33–35]. This is due to the physiological stress led by the state of pregnancy and neutrophilia [29]. The decrease in the median value of RBC count from the first to third trimester is in agreement with studies conducted in Ethiopia, Africa and Europe [33–36]. The decrease in Hgb and HCT is due to an increase in plasma volume during pregnancy is by the effect of hemodilution, hormonal changes that increases fluid retention and an increase in iron demand [29, 31]. The decrease in the median value of PLT count from first to third trimester is consistent with other findings [30, 35, 36]. This is due to the dilution effect and compensatory phenomenon by the maximal platelet destruction as the trimester progressed from the first to third trimester [36].

The study finally calculated out of range values by comparing the newly established RIs versus the company-derived values currently in use in Dire Dawa health facilities that use similar hematological analyzer. Of note, varying degrees of misclassification are noted for most hematologic parameters. This highlights the need for locally established RI. For instance, as indicated in Table 2, the lower limit RI of our finding for WBC, Gran#, Gran% and Lymph% in both genders were lower, meaning individuals are unnecessarily classified as leukopenic or neutropenic while they could have been judged as normal if the current RI was utilized. The finding of low WBC and Neutrophils lower limit agrees with an earlier study in Ethiopia [23]. The current study, however, demonstrated higher lower limit for RBC count and Lymph #; and higher in both upper and lower limit for PLT count than the currently in use RI.

Taken together, the observed variations between the RIs newly established for Dire Dawa adult male, female and pregnant women and the other studies as well as company-derived values could be attributed to several factors. These include altitudinal difference, dietary pattern, equipment type, epidemiology of different diseases (although all claimed apparently healthy population at the time of the respective studies), and criteria for selection of study population.

The current study has its own limitation in that stool examination for intestinal parasite detection and stool occult blood test were not performed. However, participants negative for the inflammatory marker CRP were included and the study adhered to follow strict study protocol that encompass all the potential exclusion criteria stated in the CLSI C28-A2 [9]. Moreover, data were collected from a more representative demographic population with a broader age distribution ensuring adequate sample size for RI determination.

## Conclusions

The finding demonstrated statistically significant difference (p<0.05) for most of hematologic parameters based on gender as well as between pregnant and non-pregnant women. This extensive variation provides evidence for the importance of utilizing the gender and pregnancy specific hematologic RI. It is vital to understand changes in hematologic parameters during pregnancy based on their gestational age to avoid pregnancy related hematologic complication. In addition, the study also adds to the growing body of knowledge concerning the effect of altitude on red cell parameters that we found lower than other studies conducted in different part of the country. This needs caution in utilizing similar RIs for highland and lowland dwellers. Moreover, the RI obtained from this study differs from the clinical practice currently utilized in Dire Dawa, Ethiopia, other African countries as well as the western population. It underscores the need for utilising locally derived hematologic RIs for better management, diagnosis and monitoring of hematologic disorders for adults of both genders and pregnant women.

### Recommendation

The reference values presented here should be used as a guide to all health facilities of Dire Dawa town for the better management, diagnosis and monitoring of hematologic disorders for adults of both genders and pregnant women. More research is needed to better understand the variation across geriatric and pediatrics age groups.
